The article "Characterization of Tumor Mutation Burden-Based Gene Signature and Molecular Subtypes to Assist Precision Treatment in Gastric Cancer" was retracted in 2024. Reasons: suspected computer-generated content; unreliable results or conclusions; concerns about the data; concerns about the results or conclusions.

# Characterization of Tumor Mutation Burden-Based Gene Signature and Molecular Subtypes to Assist Precision Treatment in Gastric Cancer

**DOI:** 10.1155/2022/4006507

**Published:** 2022-05-13

**Authors:** Cheng Wei, Minzhe Li, Shaofeng Lin, Jun Xiao

**Affiliations:** ^1^Department of Gastrointestinal Surgery, Fujian Medical University Cancer Hospital, Fujian Cancer Hospital, Fuzhou 350014, Fujian, China; ^2^General Surgery Department, Beijing Chao-Yang Hospital, Capital Medical University, Beijing 100020, China; ^3^Department of Thoracic Surgery, Fujian Medical University Cancer Hospital, Fujian Cancer Hospital, Fuzhou 350014, Fujian, China

## Abstract

**Objective:**

Tumor mutation burden (TMB) represents a useful biomarker for predicting survival outcomes and immunotherapy response. Here, we aimed to conduct TMB-based gene signature and molecular subtypes in gastric cancer.

**Methods:**

Based on differentially expressed genes (DEGs) between high- and low-TMB groups in TCGA, a LASSO model was developed for predicting overall survival (OS) and disease-free survival (DFS). The predictive performance was externally verified in the GSE84437 dataset. Molecular subtypes were conducted via consensus clustering approach based on TMB-related DEGs. The immune microenvironment was estimated by ESTIMATE and ssGSEA algorithms.

**Results:**

High-TMB patients had prolonged survival duration. TMB-related DEGs were distinctly enriched in cancer- (MAPK, P53, PI3K-Akt, and Wnt pathways) and immune-related pathways (T cell selection and differentiation). The TMB-based gene model was developed (including MATN3, UPK1B, GPX3, and RGS2), and high-risk score was predictive of poor prognosis and recurrence. ROC and multivariate analyses revealed the well predictive performance, which was confirmed in the external cohort. Furthermore, we established the nomogram containing the risk score, age, and stage for personalized prediction of OS and DFS. High-risk score was characterized by high stromal score, increased immune checkpoints, immune cell infiltrations, and enhanced sensitivity to gefitinib, vinorelbine, and gemcitabine. Three TMB-based molecular subtypes were conducted, characterized by distinct prognosis, immune microenvironment, and drug sensitivity.

**Conclusion:**

Collectively, we established a prognostic signature and three distinct molecular subtypes based on TMB features for gastric cancer, which might be beneficial for prognostic prediction and clinical decision-making.

## 1. Introduction

Gastric cancer represents a commonly diagnosed malignancy, possessing high incidence, and mortality, especially in East Asian countries [1]. It represents a heterogeneous malignancy due to morphological and phenotypic characteristics as well as geographical discrepancies [2]. The initiation and progression of gastric cancer is an intricate multistep process, involving numerous genetic and epigenetic alterations [3]. Conventional risk evaluation often ignores biological heterogeneity of gastric cancer [4]. Most of gastric cancer patients diagnosed at late stages display a five-year survival rate of less than 30% [5]. Despite great efforts in improving therapeutic efficacy, patients' survival still varies widely [6]. Selection of representative gene sets for risk stratification may offer new ideas for more precise prognoses prediction and personalized therapies.

Currently, blockade of immune checkpoints with monoclonal antibodies such as nivolumab and pembrolizumab has become an emerging strategy in treating gastric cancer [7]. For instance, clinical trials of anti-PD-1/PD-L1 therapies have displayed sustained anticancer responses and prolonged survival duration in gastric cancer [8]. However, predictive factors of immunotherapy remain systematically undefined. Genomic mutations are the major cause of gastric cancer initiation and progression [9]. Tumor mutation burden (TMB) represents the entire number of somatic protein-coding base substitutions. It has been estimated that elevated TMB is investigated in 20% of gastric cancer patients [10]. Increased TMB is a useful biomarker in predicting enhanced overall survival and benefit to anti-PD-1/PD-L1 immunotherapy in gastric cancer [8]. Nevertheless, little research has dissected prognostic implications of TMB and its relationships with immune microenvironment in gastric cancer. This study constructed TMB-related gene signature and molecular subtypes that may accurately estimate survival outcomes and drug sensitivity and reflect immune microenvironment of gastric cancer, which might assist therapeutic customization as well as clinical decision-making.

## 2. Materials and Methods

### 2.1. Data Acquisition

Somatic mutation data and transcriptome profiles of gastric cancer were retrieved from the Cancer Genome Atlas (TCGA) through the GDC data portal (https://portal.gdc.cancer.gov/). Meanwhile, matched clinical data were also downloaded from TCGA. Microarray expression profiling of 433 gastric cancer specimens was obtained from the GSE84437 dataset in the Gene Expression Omnibus (GEO; https://www.ncbi.nlm.nih.gov/geo/) database [11].  Table 1 listed clinical characteristics of TCGA and GSE84437 datasets.

### 2.2. TMB Score Calculation

TMB represents the total amount of somatic missense mutations in a tumor specimen. Here, TMB score was determined as the amount of mutations/length of exons (30 Mb) for gastric cancer specimens. Following dividing subjects into two groups based on the median value of TMB score, somatic mutation was analyzed and visualized via maftools package [12]. Overall survival (OS) difference between groups was evaluated by Kaplan-Meier curves as well as log-rank test. The distribution of TMB score was analyzed in different subgroups according to clinicopathologic features, as follows: age (≤60, >60), gender (female, male), grade (G1, G2, and G3), T stage (T1, T2, T3, and T4), M stage (M0, M1), and stage (stage I, stage II, stage III, and stage IV).

### 2.3. Differentially Expressed Gene (DEG) Screening

To determine DEGs, gene expression between high and low TMB groups was compared via limma package [13]. Genes with ∣fold − change | >1.5 and false discovery rate (FDR) < 0.05 were considered as TMB-related DEGs. Among them, genes with fold − change > 1.5 were upregulated in high TMB samples and those with fold − change < −1.5 were downregulated in high TMB samples.

### 2.4. Targeted Drug Prediction

Drug sensitivity data of Connectivity Map (CMap) drug database (http://www.broadinstitute.org/cmap) were applied for discovering small molecule drugs related to gastric cancer [14]. Up- and downregulated TMB-related genes were separately uploaded into the database and connectivity score (-1~1) was calculated. Positive connectivity score demonstrated that the gene signature was induced by this small compound, and negative score represented that the gene signature was suppressed by this compound. Here, potential small compounds were screened based on ∣connectivity score | >0.70 and *p* value < 0.05.

### 2.5. Functional Enrichment Analyses

Gene Ontology (GO) analysis of DEGs was presented utilizing clusterProfiler package [15]. GO categories contained biological process (BP), cellular component (CC), and molecular function (MF). The Kyoto Encyclopedia of Genes and Genomes (KEGG) pathways were analyzed when TMB score as a phenotype utilizing gene set enrichment analysis (GSEA) v3.0 software [16]. The reference gene set (http://c5.bp.v6.2.symbols.gm) was retrieved from the Molecular Signatures Database (http://software.broadinstitute.org/gsea/msigdb/) [17]. Terms with FDR < 0.05 were significantly activated in high or low TMB samples.

### 2.6. Establishment of a Prognostic Model

Univariate analyses were presented to assess the associations between TMB-related DEGs and survival outcomes in TCGA cohort. Genes with *p* value < 0.05 were screened for least absolute shrinkage and selection operator (LASSO) analysis. Tenfold cross-verification was employed for acquiring candidate variables. These variables with nonzero regression coefficients were utilized for multivariate analysis. The risk score was conducted by combining expression and regression coefficient of each variable. The formula was as follows: risk score = ∑_*i*=1_^*N*^(coefi∗expri). The LASSO model was established by glmnet package [18]. The risk score of each patient was calculated. Then, we stratified these patients into two groups according to the median value of risk score. The distribution of survival status was assessed in two groups. OS and disease-free survival (DFS) analyses were conducted by survminer package. Expression profiles of genes in this model were visualized into heatmap. Receiver-operator characteristic (ROC) curve analyses of OS and DFS were conducted to estimate the predictive potency utilizing survivalROC package, followed by calculation of area under the curve (AUC). The survival duration was compared with log-rank test. Furthermore, this model was externally verified in the GSE84437 cohort. By univariate analyses, associations between survival outcomes and age, gender, grade, stage, and risk score were evaluated in TCGA cohort. Multivariate analysis was further utilized for evaluating whether the parameters independently predicted patients' OS and DFS.

### 2.7. Establishment and Assessment of a Nomogram

Independent prognostic variables were included for creating a nomogram to predict one-, three-, and five-year OS and DFS of gastric cancer patients utilizing rms package in TCGA cohort. To evaluate the predictive performance of this nomogram, nomogram-predicted and actual one-, three-, and five-year OS and DFS probabilities were compared through calibration plots.

### 2.8. Evaluation of Correlation between Risk Score and Immune Microenvironment

Immune microenvironment was evaluated according to immune cell infiltrations and immune checkpoint expression. Infiltration levels of stromal and immune cells were inferred in gastric cancer specimens from TCGA cohort utilizing Estimation of Stromal and Immune Cells in Malignant Tumors using Expression data (ESTIMATE) algorithm on the basis of gene expression data [19]. Then, stromal, immune, and ESTIMATE scores were determined for each specimen. The abundances of activated B cell, activated CD4 T cell, activated CD8 T cell, central memory CD4 T cell, central memory CD8 T cell, effector memory CD4 T cell, effector memory CD8 T cell, gamma delta T cell, immature B cell, memory B cell, regulatory T cell, T follicular helper cell, type 1 T helper cell, type 17 T helper cell, type 2 T helper cell, activated dendritic cell, CD56 bright natural killer cell, CD56dim natural killer cell, eosinophil, immature dendritic cell, macrophage, mast cell, MDSC, monocyte, natural killer cell, natural killer T cell, neutrophil, and plasmacytoid dendritic cell were estimated in each sample via single-sample gene set enrichment analysis (ssGSEA) algorithm. Also, immune checkpoints were also assessed, including ADORA2A, BTLA, BTNL2, CD160, CD200, CD200R1, CD244, CD27, CD274, CD276, CD28, CD40, CD40LG, CD44, CD48, CD70, CD80, CD86, CTLA4, HAVCR2, HHLA2, ICOS, ICOSLG, IDO1, IDO2, KIR3DL1, LAG3, LAIR1, LGALS9, NRP1, PDCD1, PDCD1LG2, TIGIT, TMIGD2, TNFRSF14, TNFRSF18, TNFRSF25, TNFRSF4, TNFRSF8, TNFRSF9, TNFSF14, TNFSF15, TNFSF18, TNFSF4, TNFSF9, VSIR, and VTCN1.

### 2.9. Drug Sensitivity Analysis

The half maximal inhibitory concentration (IC50) of drugs (sorafenib, gefitinib, vinorelbine, and gemcitabine) of gastric cancer specimens was estimated based on the Genomics of Drug Sensitivity in Cancer (GDSC; http://www.cancerrxgene.org/) [20] utilizing pRRophetic package [21].

### 2.10. Consensus Clustering Analysis

ConsensusClusterPlus package was adopted for consensus clustering analysis based on the expression profiling of TMB-related DEGs [22]. The consensus heatmap and cumulative distribution function (CDF) were conducted for evaluating the optimal *k* value (ranging from 2 to 10). The procedure was repeated 500 times to ensure the reproducibility of the results.

### 2.11. Statistical Analyses

Statistical analyses were achieved through R software (v3.4.1; https://www.r-project.org/) and appropriate packages. Comparisons between two groups were estimated with Student's *t* test or Wilcoxon rank-sum test. Comparisons between three groups were conducted via Kruskal-Wallis tests. *p* value < 0.05 was set as the threshold.

## 3. Results

### 3.1. TMB Links to Prognosis and Age of Gastric Cancer

From TCGA database, we retrieved somatic mutation data of 433 gastric cancer patients. Following calculating TMB score, we separated these patients into two groups according to the median value of TMB score. Oncoplots visualized the somatic mutated landscape of high and low TMB cohorts (Figures 1(a) and 1(b)). We found the higher mutated frequency in high than low TMB samples. To compare survival duration between groups, OS analysis was carried out. Our data suggested that high TMB subjects had prolonged OS time (*p* = 0.01515; Figure 1(c)). This indicated that increased TMB might contribute to optimistic prognosis. Associations of TMB score with clinicopathological characteristics were further evaluated in gastric cancer. Only age was significantly linked to TMB score. Higher TMB score was found in patients with age > 65 compared to those with age ≤ 65 (*p* < 0.001; Figure 1(d)).

### 3.2. Screening DEGs between High and Low TMB Score

To screen TMB-related DEGs, we analyzed the difference in expression profiling between high (*n* = 191) and low (*n* = 192) TMB groups utilizing limma package. As a result, 122 genes with fold‐change > 1.5 and FDR < 0.05 were upregulated in high than low TMB groups (Figure 2(a)).  Table 2 listed the first 20 upregulated genes, as follows: C8G, LEFTY1, HOXA9 PIWIL1, HOXA11, SEMG1, NXPH4, TNFSF9, GPA33, SPDYC, PPP1R1B, CT83, ZIC2, HOXA10, CDC6, HOXA13, RPL22L1, C2CD4A, and EFNA3. Moreover, 967 downregulated genes were identified in high compared to low TMB groups (Figure 2(b)). The first 20 downregulated genes contained ALB, CYP17A1, EZHIP, APOA1, ECRG4, SMYD1, VIP, FGA, ORM1, CNN1, CASQ2, ACTG2, DES, FGG, SMPX, MYH11, SYNM, HSPB6, TACR2, and PGA5 (Table 3).

### 3.3. Prediction of Potential Targeted Drugs against Gastric Cancer Based on TMB

To ascertain potential drugs against gastric cancer, CMap analysis was presented based on TMB-related DEGs. With | connectivity score | >0.7 and *p* < 0.05, 27 candidate drugs were predicted (Table 4). Moreover, their mechanisms were further assessed, such as cytokine production inhibitor, calmodulin antagonist, and Rho-associated kinase inhibitor (Figure 2(c)).

### 3.4. Biological Functions of TMB-Related DEGs

To explore biological functions of TMB-related DEGs, we presented GO enrichment analysis. As a result, TMB-related DEGs were primarily linked to immune biological processes like chemokine-mediated pathway, lymphocyte migration, T cell selection, and T cell differentiation (Figure 3(a)). GSEA results showed that MAPK (nominal enrichment score (NES) = −0.44864, FDR = 0.005015), pathway in cancer (NES = −0.42543, FDR = 0.003), PI3K-Akt (NES = −0.47217, FDR = 0.001003), and Wnt pathways (NES = −0.49361, FDR = 0.004154) were distinctly activated in low TMB gastric cancer samples (Figure 3(b)). Meanwhile, p53 pathway activation was found in high TMB samples (NES = 1.5633, FDR = 0.047662).  Figure 3(c) showed that DEGs ACVR1, BMP6, DCN, FBN1, FMOD, FST, GREM1, GREM2, ID4, LEFTY1, LTBP1, RGMA, SMAD9, TGFB2, TGFB3, THBS1, and THSD4 were distinctly enriched in TGF-beta pathway. DAAM2, FOSL1, FZD4, FZD7, MMP7, NFATC4, PRICKLE2, PRKCB, ROR1, ROR2, RSPO3, SERPINF1, SFRP1, SFRP4, SFRP5, SOX17, TCF7L1, WNT2B, and WNT9A were significantly enriched in Wnt pathway. Also, AKT3, AREG, CACNA1C, CACNA1H, CACNA2D1, DUSP1, EFNA3, FGF2, FGF7, FGFR1, FLNA, FLNC, HGF, HSPA2, IGF1R, IL1R1, KIT, MAP3K20, MEF2C, MRAS, NGFR, PDGFD, PDGFRA, PLA2G4C, PRKCB, RASGRP2, TEK, TGFB2, and TGFB3 were enriched in MAPK pathway.

### 3.5. A TMB-Related Gene Model for Predicting Gastric Cancer Patients' OS

Univariate analyses were further conducted to determine prognostic TMB-related DEGs in gastric cancer. Among TMB-related DEGs, 436 displayed distinct relationships to survival outcomes of gastric cancer (all *p* value < 0.05; Supplementary Table 1). By applying LASSO method with 10-fold cross-verification followed by 1,000-time iterations, a 4-gene model (MATN3, UPK1B, GPX3, and RGS2) was conducted in TCGA cohort (Figures 4(a) and 4(b)). The risk score was determined by combining expression and regression coefficient of genes (MATN3: 0.0649094697586887, UPK1B: 0.0335931553068305, GPX3: 0.00612329324773029, and RGS2: 0.0128435908595123). To investigate relationships between risk score and patients' survival, we classified patients into two groups according to the median value of risk score (Figure 4(c)). High-risk group had more death cases than low-risk group (Figure 4(d)). OS analysis between groups was than conducted. Consequently, pessimistic OS duration was investigated in high- than low-risk groups (*p* value = 1.087*e*-07; Figure 4(e)). As shown in Figure 4(f), MATN3, UPK1B, GPX3, and RGS2 were all upregulated in high- compared to low-risk specimens. Through ROC analyses, the accuracy of this model was evaluated. AUC value of OS time was 0.742, indicative of the powerful prognostic prediction usefulness (Figure 4(g)).

### 3.6. This TMB-Based Gene Signature Can Accurately Predict Gastric Cancer Recurrence

We also evaluated the relationships between risk score and gastric cancer recurrence. With the same regression coefficients of genes, we stratified patients into two groups (Figure 5(a)). High-risk group had more recurred or dead cases compared to low-risk group (Figure 5(b)). In Figure 5(c), high-risk subjects displayed worse DFS than low-risk subjects (*p* value = 5.519*e*-07). The upregulation of these genes in this model was found in high- than low-risk groups (Figure 5(d)). AUC value of DFS time was 0.67, indicating that this model was capable of evaluating gastric cancer recurrence (Figure 5(e)). Our multivariate analysis confirmed that this TMB model can be independently predictive of prognosis and recurrence of gastric cancer (Figure 5(f)).

### 3.7. Validation of This TMB-Based Gene Signature in an External Cohort

To verify whether this model was credible, the external cohort (GSE84437) was utilized, which contained 433 gastric cancer patients. Following the same formula, we determined the risk score of each specimen. These subjects were stratified into high- and low-risk groups (Figure 6(a)). More dead cases were observed in high- than low-risk groups (Figure 6(b)). Heatmap visualized expression profiling of 4 genes in the GSE84437 cohort (Figure 6(c)). Poorer prognosis was found in high-risk samples (*p* value = 1.762*e*-03; Figure 6(d)). ROC analysis confirmed the accuracy as AUC = 0.628 (Figure 6(e)).

### 3.8. Establishment and Assessment of a Nomogram Model for Predicting Prognosis and Recurrence

To determine independent prognostic factors of gastric cancer, we conducted multivariate analysis. As a result, age, stage, and risk score were independently linked to gastric cancer prognosis. For systematically predicting gastric cancer prognosis and recurrence, a nomogram model was established based on above factors (Figures 7(a) and 7(b)). The calibration plots demonstrated that the model-predicted one-, three-, and five-year OS time was highly consistent with actual OS time (Figures 7(c)–7(e)). Moreover, the excellent concordance was also found between predicted one-, three-, and five-year DFS and actual DFS probabilities (Figures 7(f)–7(h)).

### 3.9. This TMB-Related Gene Model Is in relation to Immune Microenvironment and Drug Sensitivity of Gastric Cancer

To explore relationships between risk score and immune microenvironment, we evaluated immune/stromal scores and tumor purity of gastric cancer specimens in TCGA cohort. Higher stromal score was detected in high- than low-risk groups (*p* value < 0.0001; Figure 8(a)). Meanwhile, low-risk samples were characterized by increased tumor purity (*p* value < 0.001). Most of immune checkpoints were highly expressed in high- than low-risk groups, including ADORA2A, CD200, CD200R1, CD27, CD28, CD40, CD40LG, CD48, NRP1, TNFRSF4, TNFRSF8, TNFSF14, TNFSF15, TNFSF18, TNFSF4, VSIR, and VTCN1 (Figure 8(b)). Moreover, most of immune cells exhibited higher infiltration levels in high- compared to low-risk samples, including activated B cell, central memory CD4 T cell, central memory CD8 T cell, effector memory CD4 T cell, gamma delta T cell, immature B cell, memory B cell, regulatory T cell, T follicular helper cell, type 1 T helper cell, CD56 bright natural killer cell, eosinophil, immature dendritic cell, macrophage, mast cell, monocyte, natural killer cell, natural killer T cell, and plasmacytoid dendritic cell (Figure 8(c)). No significant difference in IC50 value of sorafenib was found between high- and low-risk groups (Figure 8(d)). But high-risk samples presented lower IC50 values of gefitinib, vinorelbine, and gemcitabine than low-risk samples (Figure 8(d)), indicating that high-risk patients might benefit from above agents.

### 3.10. Specific TMB-Based Molecular Subtypes in Gastric Cancer

Through consensus clustering analysis, we conducted three TMB-based molecular subtypes based on the expression profiling of TMB-related DEGs (Figures 9(a)–9(c)), named as C1, C2, and C3. Survival analysis uncovered that C2 subtype presented the best prognosis, followed by C1 and C3 (Figure 9(d)). C2 subtype had significantly reduced stromal and immune scores and increased tumor purity compared with C1 and C3 (Figure 9(e)). Moreover, we found that most immune checkpoints had the lowest expression in C2 subtype among three subtypes (Figure 9(f)). In Figure 9(g), C2 subtype had the lowest infiltration levels of immune cells. In Figure 9(h), C2 subtype had the highest sensitivity to gefitinib, while C3 subtype showed the lowest sensitivity to gefitinib, gemcitabine, and sorafenib. No significant difference in vinorelbine sensitivity was found among three subtypes.

## 4. Discussion

Due to histological and etiological heterogeneity, it is of difficulty for determining appropriate therapeutic modalities for gastric cancer. Accumulating evidences suggest that TMB is in relation to gastric cancer progress and patients' survival outcomes [23]. The genomic variant characteristics within gastric cancer influence its evolution and immunogenicity [24]. The tumors have developed a few coping strategies to respond to these alterations through DNA repair and replication (DRR). Zhang et al. has established a DRR-related gene signature on the basis of TMB that uncovers prognosis and immunotherapeutic response in gastric cancer [24]. Nevertheless, the TMB-based gene models and molecular subtypes remain lacking in gastric cancer. Hence, this study proposed a prognostic TMB-related gene model and subtype classification in gastric cancer. The model and subtypes displayed the well performance on estimating prognosis, recurrence, and immune cell infiltrations of gastric cancer.

TMB was quantified in gastric cancer, which represented the entire number of mutations [25]. For investigating the TMB-induced survival differences, we stratified patients into high- and low-TMB groups. Our data suggested that TMB-high gastric cancer patients displayed more favorable OS duration in comparison to TMB-low patients, as previously reported [26]. Moreover, it has been demonstrated that TMB is in relation to clinicopathological characteristics as well as immune cell infiltrations of gastric cancer [26]. For analyzing involved molecular mechanisms, gene expression alterations were identified. These dysregulated genes were mainly in relation to T cell differentiation and selection biological processes, indicating that they might affect immune response of T cells [27]. Furthermore, cancer-related pathways (MAPK, P53, PI3K-Akt, and Wnt pathways) were distinctly enriched by TMB-related DEGs. Above data demonstrated that TMB affected gastric cancer initiation as well as progress.

TMB has become a useful biomarker for indicating patients who may benefit from immunotherapy in clinical practice [25]. This study established a TMB prognostic model containing MATN3, UPK1B, GPX3, and RGS2 based on TMB-related DEGs. Previously, MATN3 was aberrantly methylated and expressed in gastric cancer and related to survival outcomes [28]. UPK1B expression was in relation to response to capecitabine and oxaliplatin and prognoses for gastric cancer patients [29]. GPX3 hypermethylation was in gastric cancer and correlated to lymph node metastases, tumor invasion depth, tumor differentiation as well as relapse [30]. RGS2 mediated gastric cancer proliferation and metastases [31]. Hence, above genes participated in gastric cancer progression and emerged as therapeutic targets. Our in-depth analysis revealed that this TMB prognostic model was accurately predictive of one-, three-, and five-year OS and DFS. By including TMB risk score, age- and stage-independent prognostic parameters, we created the nomogram in accurately predicting one-, three-, and five-year OS and DFS. Hence, this nomogram might offer convenient and credible prognosis prediction information in gastric cancer.

Immunotherapies have displayed astounding therapeutic efficacies in the minority of gastric cancer subjects [32]. Most of them experience minimal or no clinical benefits. A meta-analysis reported that the objective response rate was only 12.0% for gastric cancer treated with anti-PD-1/PD-L1 therapies [33]. Tumor immune microenvironment contains heterogenous cell components, which may affect cancer cellular behaviors [34]. Much research has demonstrated that tumor cells display altered biological behaviors by interactions with tumor immune microenvironment components [35, 36]. The special correlations between immune cells and TMB have been detected in gastric cancer [37]. Here, we observed the relationships between TMB risk score and immune microenvironment. As a result, high-risk score was characterized by high stromal score, increased immune checkpoints (ADORA2A, CD200, CD200R1, CD27, CD28, CD40, CD40LG, CD48, NRP1, TNFRSF4, TNFRSF8, TNFSF14, TNFSF15, TNFSF18, TNFSF4, VSIR, and VTCN1) and immune cell infiltrations (activated B cell, central memory CD4 T cell, central memory CD8 T cell, effector memory CD4 T cell, gamma delta T cell, immature B cell, memory B cell, regulatory T cell, T follicular helper cell, type 1 T helper cell, CD56bright natural killer cell, eosinophil, immature dendritic cell, macrophage, mast cell, monocyte, natural killer cell, natural killer T cell and plasmacytoid dendritic cell), indicating that high-risk subjects might be more likely to benefit from immunotherapy. Further investigation requires to perform for confirming the predictive efficacy on immunotherapy responses.

Gastric cancer is a highly heterogeneous malignant tumor. Therefore, it is of importance to classify gastric cancer into distinct subtypes [38]. Previously, Li and Wang identified three gastric cancer subtypes on the basis of the activities of pathways related to immune, DNA repair, oncogenic, and stromal signatures [38]. However, a classification of gastric cancer based on TMB remains lacking. Herein, based on the expression profiles of TMB-related DEGs, we conducted three TMB-based molecular subtypes, characterized by distinct prognosis, immune microenvironment, and drug sensitivity, which might be applied for assisting therapeutic customization and clinical decision-making in gastric cancer. Our classification of gastric cancer on the basis of TMB features might offer novel insights into the heterogeneity in gastric cancer.

## 5. Conclusion

Collectively, survival analysis demonstrated that TMB was a useful predictive parameter in gastric cancer. Through LASSO algorithm, a TMB-related gene model related to immune microenvironment was created for robustly predicting OS and DFS of gastric cancer patients in TCGA cohort, which was externally confirmed in the GSE84437 cohort. Moreover, three distinct TMB-based molecular subtypes were characterized for gastric cancer through consensus clustering approach. The TMB-based gene model and molecular subtypes might assist identifying gastric cancer subjects more likely to benefit from immunotherapy, which provides an opportunity for personalized treatment. Nevertheless, this was a retrospective study based on clinical, genomic, and mutation data from public datasets. In our future studies, we will validate the TMB-based prognosis gene signature and molecular subtypes in well-designed, prospective, and multicenter cohorts.

## Figures and Tables

**Figure 1:** TMB links to survival outcomes and age of gastric cancer. Patients in TCGA cohort were separated into two groups according to TMB median. (a) Waterfall plots for the somatic mutation landscape of the first 20 genes in gastric cancer with high TMB. (b) Waterfall plots for the somatic mutation landscape of the first 20 genes in gastric cancer with low TMB. Mutated genes are ranked according to mutated frequency. Mutated classifications are displayed in the bottom. (c) Associations between TMB and survival duration of gastric cancer subjects. *p* value was determined by log-rank test. (d) Correlation between TMB and patients' age. *p* value was assessed with unpaired Student's *t* test.

**Figure 2:** Comparisons of differential gene expression profiling in high- and low-TMB patients. DEGs between groups were screened with | FC | >1.5 and FDR < 0.05. (a) Volcano diagram visualizing up- and downregulated genes in high-TMB than low-TMB groups. Red dots represent upregulated genes. Blue dots represent downregulated genes. (b) Heatmap depicting expression patterns of downregulated genes between groups. (c) Heatmap for mechanism of action shared by small molecular compounds identified by CMap analysis.

**Figure 3:** Biological functions of TMB-related DEGs. (a) Biological processes, cellular components, and molecular functions enriched by DEGs. (b) GSEA for activated KEGG pathways in low-TMB group. (c) A pathway enrichment network of Wnt, MAPK, and TGF-beta signaling pathways.

**Figure 4:** A LASSO model based on TMB-related DEGs links to gastric cancer patients' OS in TCGA cohort. (a) Association between log*λ* and partial likelihood deviance. 10-fold cross-verification was used for selecting the optimal parameter in the LASSO model. (b) LASSO regression coefficients for genes in the model. (c) TMB risk score distribution. Vertical dotted line represented the risk score median. Patients were stratified into high- and low-risk groups. Red was indicative of high-risk group and green was indicative of low-risk group. (d) Survival status (green: alive; red: dead) distribution. (e) OS probabilities for high- and low-risk groups. *p* value was assessed via log-rank test. (f) Heatmap for expression profiles of 4 genes in this model. (g) ROC curve of OS in TCGA cohort.

**Figure 5:** The LASSO model accurately predicts gastric cancer recurrence in TCGA cohort. (a) Risk score distribution. (b) Survival status distribution. Red: recurred or dead status and green: disease free status. (c) DFS probabilities for high- and low-risk groups. *p* value was assessed via log-rank test. (d) Heatmap for expression profiling of 4 genes. (e) ROC of DFS in TCGA cohort. (f) Multivariate analysis for assessing the independence of risk score in predicting OS and DFS. HR: hazard ratio; CI: confidence interval.

**Figure 6:** External verification of this TMB-related gene model. (a–c) Distributions of risks core, survival status and expression profiles in the external cohort. (d) OS probabilities of high- and low-risk patients. *p* value was assessed with log-rank test. (e) ROC of OS in the external cohort.

**Figure 7:** A nomogram for predicting prognosis and recurrence. (a) The nomogram containing age, stage, and risk score for assessing one-, three-, and five-year OS probabilities. (b) The nomogram for assessing one-, three-, and five-year DFS probabilities. (c–e) Calibration curves of nomogram-predicted and actual one-, three-, and five-year OS probabilities. (f–h) Calibration curves of nomogram-predicted and actual one-, three-, and five-year DFS probabilities.

**Figure 8:** Association between TMB-related risk score and immune microenvironment of gastric cancer. (a) Distributions of stromal/immune scores and tumor purity in high- and low-risk groups. (b) Expression levels of immune checkpoints in two groups. (c) Infiltration levels of immune cells in two groups. (d) IC50 values to sorafenib, gefitinib, vinorelbine, and gemcitabine in two groups. *p* values were determined by Wilcoxon rank-sum tests. Ns: not significant; ^∗^*p* value < 0.05; ^∗∗^*p* value < 0.01; ^∗∗∗^*p* value < 0.001.

**Figure 9:** Specific TMB-based molecular subtypes in gastric cancer. (a) Consensus clustering matrix for *k* = 3. (b) Consensus cumulative distribution function (CDF) curves when *k* ranged from 2 to 9. (c) Relative change in area under CDF curve when *k* ranged from 2 to 9. (d) OS probabilities for three TMB-based molecular subtypes. *p* value was assessed with log-rank test. (e) Stromal/immune scores and tumor purity in three subtypes. (f) Expression levels of immune checkpoints in three subtypes. (g) Infiltration levels of immune cells in three subtypes. (h) IC50 values to gefitinib, gemcitabine, sorafenib, and vinorelbine in three subtypes. ^∗^*p* value < 0.05; ^∗∗^*p* value < 0.01; ^∗∗∗^*p* value < 0.001; ^∗∗∗∗^*p* value < 0.0001.

**Table 1:** Clinical characteristics of gastric cancer patients in TCGA and GSE84437 datasets.

Clinical characteristics	TCGA dataset (*n*)	GSE84437 dataset (*n*)
Age		
≤65	155	283
>65	186	150
Gender		
Female	121	137
Male	220	296
Grade		
G1	8	
G2	116	
G3	217	
Stage		
Stage I	40	
Stage II	114	
Stage III	154	
Stage IV	33	
T		
T1	15	11
T2	70	38
T3	169	92
T4	87	292
N		
N0	105	80
N1	94	188
N2	71	132
N3	71	33
M		
M0	320	
M1	21	

**Table 2:** The first 20 upregulated genes in high-TMB than low-TMB groups.

Gene	Mean value		Logfold-change	*p* value	FDR
	Low-TMB group (*n* = 192)	High-TMB group (*n* = 191)			
C8G	1.808	7.266	2.007	0.025	0.045
LEFTY1	2.634	10.220	1.956	0.014	0.027
HOXA9	0.656	2.431	1.889	5.35*E*-08	7.06*E*-07
PIWIL1	0.645	1.805	1.485	3.07*E*-07	3.05*E*-06
HOXA11	1.131	3.092	1.451	4.48*E*-12	4.46*E*-10
SEMG1	0.842	2.247	1.416	0.008	0.018
NXPH4	1.901	4.911	1.370	0.0004	0.001
TNFSF9	3.366	8.151	1.276	0.0004	0.001
GPA33	8.997	20.799	1.209	1.71*E*-05	8.84*E*-05
SPDYC	0.934	2.124	1.185	2.67*E*-06	1.85*E*-05
PPP1R1B	32.777	72.955	1.154	1.08*E*-05	5.99*E*-05
CT83	4.971	10.594	1.092	0.0001	0.0004
ZIC2	1.603	3.400	1.085	2.78*E*-05	0.0001
HOXA10	2.724	5.693	1.063	2.24*E*-12	2.78*E*-10
CDC6	7.140	14.790	1.051	1.04*E*-07	1.22*E*-06
HOXA13	3.135	6.419	1.034	7.85*E*-09	1.48*E*-07
RPL22L1	17.473	35.002	1.002	1.53*E*-05	8.05*E*-05
C2CD4A	3.873	7.674	0.986	4.39*E*-05	0.0002
EFNA3	4.540	8.868	0.966	5.90*E*-08	7.69*E*-07

**Table 3:** The first 20 downregulated genes in high-TMB than low-TMB groups.

Gene	Mean value		Logfold-change	*p* value	FDR
	Low-TMB group (*n* = 192)	High-TMB group (*n* = 191)			
ALB	78.560	0.882	-6.477	0.004	0.009
CYP17A1	5.257	0.315	-4.062	0.0003	0.001
EZHIP	3.915	0.285	-3.783	0.003	0.007
APOA1	78.826	11.510	-2.776	0.003	0.007
ECRG4	9.257	1.402	-2.723	7.94*E*-08	9.81*E*-07
SMYD1	2.298	0.353	-2.701	0.004	0.009
VIP	4.074	0.649	-2.650	7.01*E*-05	0.0003
FGA	6.056	0.975	-2.634	0.0003	0.001
ORM1	21.500	3.575	-2.589	0.012	0.025
CNN1	149.697	25.116	-2.575	5.89*E*-06	3.60*E*-05
CASQ2	3.567	0.616	-2.533	2.05*E*-08	3.23*E*-07
ACTG2	343.749	59.775	-2.524	6.95*E*-06	4.15*E*-05
DES	601.068	107.208	-2.487	2.43*E*-05	0.0001
FGG	4.239	0.764	-2.471	0.0002	0.0006
SMPX	2.869	0.525	-2.452	0.018	0.033
MYH11	181.815	33.262	-2.451	4.08*E*-07	3.82*E*-06
SYNM	35.312	6.474	-2.447	3.07*E*-08	4.46*E*-07
HSPB6	132.416	24.497	-2.434	1.01*E*-08	1.80*E*-07
TACR2	10.288	1.909	-2.430	0.003	0.008
PGA5	7.939	1.518	-2.386	0.016	0.031

**Table 4:** CMap analysis identifies potential small molecular compounds.

CMap name	Mean	*N*	Enrichment	*p* value	Specificity	Percent nonnull
Levomepromazine	0.760	4	0.896	0.0001	0.015	100
W-13	0.469	2	0.855	0.042	0.037	100
Diethylstilbestrol	0.686	6	0.850	0.00002	0	100
Cefoperazone	0.493	3	0.842	0.008	0.005	66
Vanoxerine	0.477	4	0.823	0.002	0.010	75
Terbutaline	0.303	4	0.774	0.005	0.006	50
PF-00875133-00	0.397	3	0.769	0.024	0.006	66
Kinetin	0.316	4	0.763	0.006	0	50
Fendiline	0.414	3	0.720	0.043	0.082	66
Vinburnine	0.348	4	0.718	0.013	0.053	50
Cefixime	-0.408	4	-0.705	0.016	0.005	50
Apigenin	-0.613	4	-0.706	0.015	0.103	75
Piroxicam	-0.524	4	-0.706	0.016	0.029	75
PNU-0230031	-0.305	8	-0.721	0.0001	0.005	50
Prestwick-682	-0.258	4	-0.727	0.011	0.021	50
Megestrol	-0.365	4	-0.728	0.011	0	75
Aminoglutethimide	-0.437	3	-0.760	0.028	0.024	66
Corticosterone	-0.394	4	-0.775	0.005	0	75
Fluorometholone	-0.627	4	-0.792	0.004	0	100
Withaferin A	-0.622	4	-0.804	0.009	0.090	100
Methacholine chloride	-0.719	3	-0.837	0.009	0.026	100
5224221	-0.647	2	-0.862	0.038	0.218	100
Y-27632	-0.773	2	-0.907	0.017	0.016	100
Pargyline	-0.75	4	-0.93	0.00002	0	100
Alcuronium chloride	-0.730	2	-0.936	0.009	0	100

## Data Availability

The data used to support the findings of this study are included within the supplementary information files.

## Abbreviations

TMB: Tumor mutation burden
TCGA: The Cancer Genome Atlas
GEO: Gene Expression Omnibus
OS: Overall survival
DEG: Differentially expressed gene
FDR: False discovery rate
CMap: Connectivity Map
GO: Gene Ontology
BP: Biological process
CC: Cellular component
MF: Molecular function
KEGG: Kyoto Encyclopedia of Genes and Genomes
GSEA: Gene set enrichment analysis
LASSO: Least absolute shrinkage and selection operator
DFS: Disease-free survival
ROC: Receiver-operator characteristic
AUC: Area under the curve
ESTIMATE: Estimation of Stromal and Immune Cells in Malignant Tumors using Expression data
ssGSEA: Single-sample gene set enrichment analysis
NES: Nominal enrichment score
HR: Hazard ratio
CI: Confidence interval.

## Supplementary Materials

Supplementary Materials Supplementary Table 1: univariate analysis for prognosis-related TMB DEGs in gastric cancer.
